The article "A Novel Biomarker, FKBP10, for Poor Prognosis Prediction in Patients with Clear Cell Renal Cell Carcinoma" was retracted in 2023. Reasons: signs of a paper mill; suspected computer-generated content; unreliable results or conclusions; concerns about the data.

# A Novel Biomarker, FKBP10, for Poor Prognosis Prediction in Patients with Clear Cell Renal Cell Carcinoma

**DOI:** 10.1155/2022/5490644

**Published:** 2022-06-10

**Authors:** Yongshuang Xiao, Shuofeng Li, Meng Zhang, Xin Liu, Guanqun Ju, Jianquan Hou

**Affiliations:** ^1^Department of Urology, The First Affiliated Hospital of Soochow University, Suzhou 215006, China; ^2^Department of Urology, The Affiliated Hospital of Xuzhou Medical University, Xuzhou 221002, China

## Abstract

**Objective:**

To screen genes associated with poor prognosis of clear cell renal cell carcinoma (CcRCC) from the public databases HPA (Human Protein Atlas), UALCAN, and GEPIA (Gene Expression Profiling Interactive Analysis) and to investigate the expression of FKBP10 in CcRCC and the effect on prognosis of the patients and the biological behavior of CcRCC cells.

**Methods:**

The tumor tissues and adjacent noncancerous tissues of 42 patients with CcRCC diagnosed and treated in our hospital were collected, and the general information of the patients was recorded. FKBP10 expression in the tissues was determined by qRT-PCR and western blot, and its relationship with general information and prognosis of patients was analyzed. Knockdown or overexpression experiments were carried out with the human proximal tubule epithelial cell line HK-2 and CcRCC cell lines Caki-1, 786-O, ACHN, and A498 to verify the relationship between FKBP10 expression and cell proliferation and adhesion ability using MTT assay and fibronectin adhesion assay, respectively. Western blot was utilized to examine the protein expression level of c-Myc, cyclin D1, and Bcl-2 in the cells.

**Results:**

FKBP10 was highly expressed in CcRCC tissues and cells and was correlated with poor prognosis. In addition, FKBP10 expression was positively correlated with CcRCC tumor size and staging and negatively correlated with tumor differentiation. Moreover, knockdown of FKBP10 significantly inhibited the proliferation of CcRCC cells, notably declined the protein expression of c-Myc, cyclin D1, and Bcl-2, and promoted cell adhesion.

**Conclusion:**

FKBP10 is highly expressed in CcRCC tissues and cells and is associated with poor prognosis in patients. FKBP10 participated in the occurrence and development of CcRCC by promoting cell proliferation and inhibiting apoptosis and adhesion.

## 1. Introduction

Renal cell carcinoma (RCC), also known as renal adenocarcinoma or renal carcinoma, is originated from tubular epithelial cells. According to the statistics, RCC ranks second among all types of urinary system malignancies [1,2]. Moreover, recent research has shown that the incidence of RCC is obviously higher compared with the past [3]. Epidemiological studies have shown that RCC accounts for approximately 3% of new malignancies each year in adults, and the incidence of RCC has been increasing over the past two decades. Clear cell renal cell carcinoma (CcRCC) is the most common histological type of RCC, with an incidence of approximately 80–85% of all types of renal cancers [4]. At present, radical nephrectomy is the major treatment for RCC in clinical practice. Specifically, surgical resection is a common and effective therapeutic method for tumors confined in the perirenal fascia (Gerota fascia). However, there is still a lack of effective methods for the treatment of patients with advanced renal cancer and postoperative recurrence and metastasis of renal cancer [5,6]. Although molecular targeted therapeutic agents have been applied in the treatment of renal cancer in clinical practice, and the prognosis has also been greatly improved, the overall therapeutic effect of patients with renal cancer is still poor [7]. Due to the lack of reliable and specific diagnostic biomarkers, a distant metastasis occurs in approximately 15–17% of patients with renal cancer at the time of clinical diagnosis, resulting in a poor prognosis [8]. Therefore, there is an urgent need to find reliable biomarkers and therapeutic targets of CcRCC to enhance treatment effects and improve prognosis.

The article "A Novel Biomarker, FKBP10, for Poor Prognosis Prediction in Patients with Clear Cell Renal Cell Carcinoma" was retracted in 2023. Reasons: signs of a paper mill; suspected computer-generated content; unreliable results or conclusions; concerns about the data.

Malignant tumors have become one of the main causes endangering human health. With the deepening research of cancers and the rapid development of high-throughput detection and analysis technologies in recent years, tumor-related genomics data have grown exponentially. The application of data mining techniques for the data analysis of a great many tumor samples can contribute to the acquisition of conclusions with regularities, the exploration of features of tumorigenesis, and the clarification of the mechanism of tumor occurrence and development. All the above are difficult to be conducted through a single trial. The use of biological information technology for the collection, analysis, and storage of tumor-related data is becoming an indispensable method for tumor-related research. And high-quality tumor bioinformatics databases provide a convenient data analysis and sharing platform for researchers, further promoting the development of related research in the medical field. In this study, the databases Human Protein Atlas (HPA) [9], UALCAN [10], and Gene Expression Profiling Interactive Analysis (GEPIA) [11] were chosen to screen and obtain the target gene FKBP10. And the expression and functions of FKBP10 were verified in the tissues and cell lines of patients with CcRCC.

FKBP10, a protein located in the endoplasmic reticulum, belongs to the FKBP-type peptidyl-prolyl cis-trans isomerase (PPIase) family, which exerts functions as molecular chaperones. The FKBP10 gene, a member of FK506-binding family, is located at 17q21.2 and encodes a protein with a molecular weight of 65 kDa. FK506-binding proteins (FKBPs) are named for their ability to specifically bind the immunosuppressant FK506 (tacrolimus) [12,13]. Specifically, FKBPs bind to the FK506 to significantly inhibit the activity of peptidyl-prolyl cis/trans isomerase (PPIase) domain activity, thereby preventing Ca2+-dependent associated pathway activation [14]. In addition, in the endoplasmic reticulum of fibroblasts, the FKBP10 protein binds to Hsp47 (heat shock protein 47) to promote the synthesis of procollagen and formation of mature collagen molecules, thereby forming a more stable complex to construct extracellular matrix [15,16]. FKBP10 expression is aberrant in a variety of malignancies and is often associated with poor prognosis in patients [17,18]. It has been reported that FKBP10 expression is negatively correlated with the survival rate of lung cancer patients, and the regulative effect of FKBP10 on protein translation sustains the growth of lung cancer [12]. It has also been stated that FKBP10 overexpression can promote the occurrence of renal cancer, which is a new promising biomarker and therapeutic target for renal cancer [19]. However, the expression and role of FKBP10 in CcRCC are still unknown. Therefore, the expression of FKBP10 in CcRCC and the effect on the biological behavior of CcRCC cells were investigated through clinical samples and in vitro experiments in this study.

The article "A Novel Biomarker, FKBP10, for Poor Prognosis Prediction in Patients with Clear Cell Renal Cell Carcinoma" was retracted in 2023. Reasons: signs of a paper mill; suspected computer-generated content; unreliable results or conclusions; concerns about the data.

## 2. Materials and Methods

### 2.1. Bioinformatics Analysis

Genes associated with renal cancer prognosis were first analyzed using the cancer module of HPA (https://www.proteinatlas.org/). Then, the genes with higher expression in renal cancer in the protein expression module of the HPA website were analyzed, and FKBP10 expression in renal cancer tissues was further queried online. After that, the UALCAN-TCGA online database (http://ualcan.path.uab.edu/index.html) was utilized to analyze the differential expression of FKBP10 in renal cancer tissues and normal tissues, as well as different staging and types of renal cancers. Then, the survival analysis was also conducted with the UALCAN-TCGA online database. Further, the GEPIA database (http://gepia.cancer-pku.cn/index.html) was utilized to validate the differential expression of FKBP10 in CcRCC cells and survival of patients in the TCGA database.

### 2.2. Clinical Samples

Tumor tissues and adjacent noncancerous tissues were collected from 42 patients with CcRCC who underwent surgical resection in our hospital. And clinical information of patients was recorded, including age, gender, tumor size (≤4; >4), TNM staging (I + II; III + IV), degree of differentiation (well-differentiated; poorly differentiated), lymphatic metastasis (positive; negative), and distant metastasis (positive; negative).

The article "A Novel Biomarker, FKBP10, for Poor Prognosis Prediction in Patients with Clear Cell Renal Cell Carcinoma" was retracted in 2023. Reasons: signs of a paper mill; suspected computer-generated content; unreliable results or conclusions; concerns about the data.

Inclusion criteria were as follows: (1) patients who were diagnosed with CcRCC through clinical data, laboratory examination, and imaging examination (CT and MRI) and underwent surgical resection in our hospital from March 2015 to July 2019, and the resected tissues were diagnosed as CcRCC by Pathology Department; (2) patients who had complete medical records and at least 6 months of follow-up records. All tissues were determined as CcRCC or normal renal tissues by doctors from Pathology Department. And the patients were divided into an upregulated group and a downregulated group according to the median expression level of FKBP10 in tumor tissues. In addition, informed consent forms were signed by all patients, and this study was approved by the Ethics Committee of the Affiliated Hospital of Xuzhou Medical University (XYFY2019-KL-032-01).

### 2.3. Cell Culture

The human proximal tubule epithelial cell line HK-2 and CcRCC cell lines Caki-1, 786-O, ACHN, and A498 were purchased from the Chinese Academy of Sciences Shanghai Branch. And the cells were cultured using mixed DMEM/F12 (Invitrogen, Carlsbad, CA, USA) and 10% of fetal bovine serum (FBS; Invitrogen, Carlsbad, CA, USA) in an incubator containing 5% of CO_2_ with a temperature of 37°C.

### 2.4. Cell Transfection

FKBP10 siRNA (si-FKBP10) and its negative control (si-NC, 100 nM) and pcDNA3.1-FKBP10 (OE-FKBP10) and its negative control (OE-NC, 100 nM) were purchased from GenePharma (Shanghai, China). The transfection was performed according to the instruction of Lipofectamine 2000 reagent (Invitrogen, Carlsbad, CA, USA) when the degree of 786-O cell fusion reached 70–80%. After 6 hours of transfection, the transfection medium was replaced with a fresh one. Then, after 48 h, the subsequent trials were continued.

### 2.5. MTT

The cell suspension with the concentration of 10^5^ cell/mL was prepared by 786-O cells. Then, 100 *μ*L of cell suspension was added in each well of a 96-well cell culture plate. After that, the plate was placed in the incubator for culture. After 48 h, the plate was taken out to add 10 *μ*L of MTT solution (5 mg/mL; Invitrogen, Carlsbad, CA, USA) in each well for static culture. After 4 h, the nutrient growth substances were removed, and then 100 *μ*L of DMSO solution was added to each well to dissolve the crystallization. Subsequently, the absorbance of solution in each well at 490 nm was measured using a microplate reader.

The article "A Novel Biomarker, FKBP10, for Poor Prognosis Prediction in Patients with Clear Cell Renal Cell Carcinoma" was retracted in 2023. Reasons: signs of a paper mill; suspected computer-generated content; unreliable results or conclusions; concerns about the data.

### 2.6. qRT-PCR

The samples of cells and tissues were collected, and the total RNA was extracted using TRIzol reagent (Invitrogen, Carlsbad, CA, USA). After that, the reverse transcription of total RNA was conducted according to the instruction of the reverse transcription kit (TaKaRa, Tokyo, Japan). Then, the LightCycler 480 (Roche, Indianapolis, IN, USA) fluorescent quantitative PCR instrument was utilized to determine the expression of genes. And the reaction conditions of PCR were carried out based on the instruction of the fluorescent quantitative PCR kit (SYBR Green Mix; Roche Diagnostics, Indianapolis, IN). Three replicates were set up for each reaction of quantitative PCR, and GAPDH was utilized as an internal control. In addition, data analysis was performed using 2^−ΔΔCt^. The primer sequences utilized in this study are shown in Table 1.

### 2.7. Western Blot

After the cells were lysed using RIPA lysis solution (Beyotime Biotechnology, Shanghai, China), the centrifugation was conducted at 12000 rpm for 15 min with a temperature of 4°C to collect the supernatant and obtain protein samples. Subsequently, the BCA kit (Beyotime Biotechnology, Shanghai, China) was used for the detection of protein concentration. Then, the corresponding volume of proteins was mixed with the loading buffer (Beyotime Biotechnology, Shanghai, China). After that, a 5-minute boiling water bath was conducted for the denaturation of the proteins. Subsequently, the protein samples were separated by SDS-PAGE and then transferred into PVDF membranes. Subsequently, the membranes were placed in the blocking solution containing 5% of skimmed milk for 60-minute blocking at ambient temperature. Further, primary antibodies were added for incubation overnight at 4°C on a shaker. Specifically, the primary antibodies applied included GAPDH (5174S, 1 : 1000; Cell Signaling, Boston, USA), FKBP10 (# 92445S, 1 : 1000; Cell Signaling), c-Myc (# 18583S, 1 : 1000; Cell Signaling), cyclin D1 (# 55506S, 1 : 1000; Cell Signaling), and Bcl-2 (# 15071S, 1 : 1000; Cell Signaling). On the second day, the membranes were washed with TBST 3 times, each time for 10 min. Then, the membranes were transferred into the secondary antibody (horseradish peroxidase-labeled goat anti-rabbit IgG, 1 : 5000; Beijing ComWin Biotech Co., Ltd., Beijing, China). After that, another 1-h incubation was conducted at ambient temperature. Then, the membranes were washed 3 times, each time for 10 min. After dripping the developer on the membrane, the detection was performed using a chemiluminescence imaging system (Bio-Rad).

The article "A Novel Biomarker, FKBP10, for Poor Prognosis Prediction in Patients with Clear Cell Renal Cell Carcinoma" was retracted in 2023. Reasons: signs of a paper mill; suspected computer-generated content; unreliable results or conclusions; concerns about the data.

### 2.8. Fibronectin Cell Adhesion Assay

A 12-well plate was preplated with fibronectin for 5 *μ*g/mL and then placed at ambient temperature for 2 h. Then, 1 × 10^5^ cells were seeded into the wells plated with fibronectin. After 1-h incubation at 37°C, nonadherent cells were removed with rinsing using phosphate-buffered saline (PBS). Subsequently, the cells were fixed using 4% of paraformaldehyde for 30 min and stained with 0.2% of crystal violet for 1 min. Then, 2% sodium dodecyl sulfate (SDS) solution was applied to dissolve crystal violet (Excess crystal violet was rinsed with water). Finally, absorbance values were measured at 570 nm through a microplate reader.

### 2.9. Statistical Analysis

All experimental data were statistically analyzed using SPSS 24.0 software and were expressed in the form of mean ± standard deviation (SD). Comparisons between two or multiple groups were performed by the *t*-test or one-way ANOVA. Prognostic factors were analyzed by univariate and multivariate Cox regression. And GraphPad Prism 8.0 was adopted for graphic plotting. *P* < 0.05 suggested that the difference was statistically significant.

## 3. Results

### 3.1. The Correlation between FKBP10 Expression and the Poor Prognosis of Patients with Clear Cell Renal Cell Carcinoma

Genes associated with CcRCC were first screened by online databases. The HPA pathology atlas showed that there were 3209 genes associated with poor prognosis and 2755 genes associated with good prognosis of renal cancer (Figure 1(a)). The top 20 important genes associated with poor prognosis were further revealed, finding high FKBP10 expression (Figure 1(b)). And FKBP10 expression was significantly increased in the cytoplasm of CcRCC (Figure 1(c)). Next, we used the unpaired Student's *t*-test to verify the difference in FKBP10 expression in different subgroups. The results of the UALCAN database also showed that FKBP10 was significantly upregulated in CcRCC, and FKBP10 expression was increased with the increase of the cancer stage and tumor grade. Besides, FKBP10 expression was high in male patients, while it was lower in Asian patients (Figure 1(d)). The relationship between FKBP10 expression and patient prognosis was further analyzed. And the results showed that high FKBP10 expression was associated with the poor prognosis of patients, and high FKBP10 expression aggravated the poor prognosis in male patients, patients with high-grade tumors, and patients of different ethnic groups (Figure 1(e)). Subsequently, the data obtained from the TCGA database were further validated by unpaired Student's *t*-test using the GEPIA database. And the results of validation also displayed that FKBP10 was notably upregulated in CcRCC (Figure 1(f)), and Kaplan–Meier survival analysis indicated that FKBP10 was associated with the poor prognosis of patients (Figure 1(g)). All in all, by analyzing data from online databases, we found that FKBP10 may be a related gene for poor prognosis in CcRCC.

The article "A Novel Biomarker, FKBP10, for Poor Prognosis Prediction in Patients with Clear Cell Renal Cell Carcinoma" was retracted in 2023. Reasons: signs of a paper mill; suspected computer-generated content; unreliable results or conclusions; concerns about the data.

### 3.2. FKBP10 Expression Can Act as a Prognosis-Related Factor in Patients with Clear Cell Renal Cell Carcinoma

The patients were divided into an upregulated group and a downregulated group according to FKBP10 median expression levels in the tumor tissues. Then, the general information of patients was recorded. We used the unpaired Student's *t*-test to analyze the relationship between FKBP10 and the general information of patients. The results indicated that FKBP10 expression was associated with TNM staging, degree of differentiation, lymphatic metastasis, and distal metastasis. However, there was no significant correlation with age, gender, or tumor size (Table 2). Univariate and multivariate Cox regression analyses were further performed for prognostic factors in patients with CcRCC. The results of analyses suggested that age and gender were not prognostic factors in patients with CcRCC, while tumor size, TNM staging, degree of differentiation, lymphatic metastasis, distant metastasis, and FKBP10 expression level could act as prognostic factors in patients with CcRCC. The results of the further multivariate analysis revealed that tumor size and distant metastasis were not prognostic factors in patients with CcRCC, while the degree of differentiation, TNM staging, lymphatic metastasis, and FKBP10 expression level could work as prognostic factors in patients with CcRCC (Table 3).

### 3.3. High FKBP10 Expression in the Cells of Patients with Clear Cell Renal Cell Carcinoma

FKBP10 expression in the tissues of CcRCC patients were further examined through qRT-PCR, and differences of FKBP10 expression in different tumor sizes, stages, and differentiation were analyzed. The results suggested that both mRNA and protein expression of FKBP10 were obviously increased in tumor tissues compared with the normal group (Figures 2(a) and 2(b)). Besides, FKBP10 expression was significantly higher in tissues with tumors >4 cm than in tissues with tumors ≤4 (Figure 2(c)). And FKBP10 expression was significantly higher in tissues with III + IV staging than in those with I + II staging (Figure 2(d)). Further, FKBP10 expression was notably higher in poorly differentiated tissues than in well-differentiated tissues (Figure 2(e)). The above results indicated that high FKBP10 expression was associated with malignant development of CcRCC. In addition, FKBP10 expression was significantly higher in CcRCC cell lines Caki-1, 786-O, ACHN, and A498 than in normal cells, and FKBP10 expression was highest in 786-O (Figure 2(f)). Therefore, 786-O cells were selected for subsequent functional experiments. In conclusion, FKBP10 was highly expressed in tissues and cell lines of patients with CcRCC and had a positive correlation with tumor size and stage and a negative correlation with tumor differentiation.

The article "A Novel Biomarker, FKBP10, for Poor Prognosis Prediction in Patients with Clear Cell Renal Cell Carcinoma" was retracted in 2023. Reasons: signs of a paper mill; suspected computer-generated content; unreliable results or conclusions; concerns about the data.

### 3.4. Knockdown of FKBP10 Inhibits the Malignant Progression of Clear Cell Renal Cell Carcinoma Cells

After further knockdown or overexpression of FKBP10, FKBP10 expression in cells was examined using qRT-PCR. The result of examination showed that FKBP10 expression in cells was correspondingly decreased or increased after knockdown or overexpression of FKBP10 (Figure 3(a)), suggesting successful cell transfection. In addition, knockdown of FKBP10 significantly reduced cell proliferation and cell adhesion ability, and the opposite was shown after overexpression of FKBP10 (Figures 3(b) and 3(c)). The protein expression level of c-Myc, cyclin D1, and Bcl-2 was notably decreased in cells after knockdown of FKBP10 and was significantly increased after overexpression of FKBP10 (Figure 3(d)). All in all, knockdown of FKBP10 promoted apoptosis and inhibited cell proliferation and adhesion ability in CcRCC cells, and vice versa.

## 4. Discussion

CcRCC, accounting for 70%–80% of all renal cancers, is the most common and most malignant RCC [20]. Therefore, it is of great significance to research the occurrence and development of CcRCC. In recent years, due to the booming development of the field of life sciences, an increasing number of researchers have begun to explore the genetic characteristics and the possible biological markers of the disease, which will provide a better basis for the diagnosis and treatment of CcRCC. With the continuous discovery of new biological markers, corresponding targeted drugs are also emerging, which are gradually becoming one of the important options for the treatment of advanced renal cancer.

It has been widely reported that fibroblast FKBP10 is expressed at a higher level in idiopathic pulmonary fibrosis tissue compared with normal lung tissue, while knockdown of FKBP10 can reduce the synthesis of collagen and reduce the migration of fibroblasts [21]. Also, some studies have found higher expression levels of FKBP10 in CcRCC tissues than in normal tissues [22]. In addition, it has been found that FKBP10 can be used as a new biomarker for bioinformatics analysis and in vitro experiments of gastric cancer prognosis and lymphatic metastasis [18]. Liang et al. [17] also demonstrated that FKBP10 is upregulated in gastric cancer tissues and is associated with worse prognosis. FKBP10 may be involved in the development of gastric cancer through cell adhesion molecules and extracellular matrix-receptor interaction pathways, and FKBP10 may be a potential therapeutic target for the treatment of gastric cancer. In this study, we found that FKBP10 expression was significantly upregulated in CcRCC tissues compared with adjacent noncancerous tissues and was correlated with poor prognosis in CcRCC patients. According to the data from public databases, the same results were obtained by qRT-PCR and western blot experiments. Besides, high FKBP10 expression could promote proliferation of CcRCC cells.

The article "A Novel Biomarker, FKBP10, for Poor Prognosis Prediction in Patients with Clear Cell Renal Cell Carcinoma" was retracted in 2023. Reasons: signs of a paper mill; suspected computer-generated content; unreliable results or conclusions; concerns about the data.

The PI3K/AKT signaling pathway is an important pathway that transmits extracellular signals into the nucleus, which plays an important regulatory role in cell proliferation, apoptosis, survival, metabolism, and other life activities. Apoptosis, a physiological form of cellular autodestruction to ensure the normal development of multicellular organisms, is the key to maintaining the balance of body tissues and the stability of the internal environment. Besides, apoptosis resistance is one of the important characteristics of tumors. Studies of various antitumor drugs have revealed that the inhibition of the PI3K/Akt signaling pathway activation can induce cell-cycle arrest and apoptosis of tumors, thereby achieving effects of tumor suppression [23]. In gastric cancer, FKBP10 promotes the PI3K/AKT signaling pathway to affect the cell viability, colony-forming ability, migration, and invasive potential of gastric cancer cells [13]. In this study, we found that FKBP10 could promote cell proliferation by affecting the protein expression of c-Myc and cyclin D1 (cell cycle-related genes of PI3K/AKT pathway downstream) in cells. In addition, we studied mitochondrial apoptosis pathway-related proteins after knockdown or overexpression of FKBP10. The results of the study indicated that FKBP10 could regulate apoptosis by affecting BLC-2 expression. In conclusion, overexpression of FKBP10 in CcRCC can affect the protein expression of c-Myc and cyclin D1 (cell cycle-related genes of PI3K/AKT pathway downstream) in cells to promote cell proliferation. Besides, FKBP10 can affect the expression of mitochondrial apoptosis pathway-related protein BCL-2 to regulate apoptosis.

## 5. Conclusion

In summary, FKBP10 can act as a prognostic marker for the patients with CcRCC. And low FKBP10 expression can affect the proliferation, adhesion, apoptosis, and other proceedings of CcRCC cells.

## Figures and Tables

**Figure 1:** Online database analysis of the relationship between FKBP10 expression and the prognosis of patients with clear cell renal cell carcinoma. (a) HPA database displayed genes associated with renal cancer prognosis. The red bars represent oncogenes, and the green bars represent suppressor genes. (b) HPA database showed the top 20 genes associated with poor prognosis of renal cancer. (c) HPA database showed FKBP10 expression in clear cell renal cell carcinoma (CcRCC) tissues and normal tissues. (d) UALCAN database revealed the FKBP10 expression level in patients with different types of CcRCC, ^*∗∗*^*P* < 0.01 vs. normal, #*P* < 0.05 vs. male; &*P* < 0.05 vs. Caucasian. (e) UALCAN database showed the relationship between FKBP10 expression and the survival analysis of patients with different types of CcRCC. (f) GEPIA database displayed FKBP10 expression in patients with CcRCC. Red indicates the CcRCC tumor group, and gray indicates the normal control group; ^*∗*^*P* < 0.05 vs. normal. (g) GEPIA database revealed the association between FKBP10 expression and the survival curve of patients with CcRCC.

The article "A Novel Biomarker, FKBP10, for Poor Prognosis Prediction in Patients with Clear Cell Renal Cell Carcinoma" was retracted in 2023. Reasons: signs of a paper mill; suspected computer-generated content; unreliable results or conclusions; concerns about the data.

**Figure 2:** FKBP10 expression in tissues and cell lines of patient with clear cell renal cell carcinoma, FKBP10 expression in tissues was checked through qRT-PCR (a) and western blot (b), ^*∗∗*^*P* < 0.01 vs. normal. QRT-PCR was utilized to determine FKBP10 expression in tumors with different sizes (c), ^*∗∗*^*P* < 0.01 vs. ≤4 group; staging (d), ^*∗∗*^*P* < 0.01 vs. stage III + IV; degree of differentiation (e), ^*∗∗*^*P* < 0.01 vs. well-differentiated; and in different cells (f), ^*∗∗*^*P* < 0.01 vs. HK-2 cell.

**Figure 3:** Effect of knockdown of FKBP10 on malignant progression of clear cell renal cell carcinoma cells. (a) FKBP10 expression in cells was determined using qRT-PCR. (b) MTT assay was performed to test cell proliferation ability in each group. (c) Fibronectin cell adhesion assay was conducted to check the adhesion ability of the cells. (d) Western blot was for the detection of the expression of c-Myc, cyclin D1, and Bcl-2 in cells. ∗∗*P* <0.01 vs. si-NC; ##*P* < 0.01 vs. OE-NC.

**Table 1:** Primer sequences.

Primer		Sequence (5′-3′)
FKBP10	Forward	CGCTACCACTACAATGGCTCCT
	Reverse	GATGTAACCCTGCCCGATATAGG
GAPDH	Forward	GGAGCGAGATCCCTCCAAAAT
	Reverse	GGCTGTTGTCATACTTCTCATGG

**Table 2:** General information of patients.

Features	Total	FKBP10 upregulated group (*n* = 22)	FKBP10 downregulated group (*n* = 20)	*P* value
Age (years)				0.662
≤55	28	14	14	
>55	14	8	6	
Gender				0.537
Male	21	12	9	
Female	21	10	11	
Tumor size (cm)				0.014
≤4	19	6	13	
>4	23	16	7	
TNM staging				0.005^*∗∗*^
I + II	22	7	15	
III + IV	20	15	5	
Degree of differentiation				0.014^*∗*^
Well-differentiated	19	6	13	
Poorly differentiated	23	16	7	
Lymphatic metastasis				0.001^*∗∗∗*^
Positive	13	12	1	
Negative	29	10	19	
Distant metastasis				0.018^*∗*^
Positive	8	7	0	
Negative	24	15	20	

^*∗*^ *P* < 0.05, ^*∗∗*^*P* < 0.01, and ^*∗∗∗*^*P* < 0.001; downregulated group vs. upregulated group.

The article "A Novel Biomarker, FKBP10, for Poor Prognosis Prediction in Patients with Clear Cell Renal Cell Carcinoma" was retracted in 2023. Reasons: signs of a paper mill; suspected computer-generated content; unreliable results or conclusions; concerns about the data.

**Table 3:** Univariate and multivariate Cox regression analyses of CcRCC prognostic factors.

Factors	Univariate Cox regression analysis			Multivariate Cox regression analyses		
	HR	95% CI	*P* value	HR	95% CI	*P* value
Age	0.896	0.675–1.238	0.268			
Gender	0.956	0.556–1.069	0.167			
Tumor size	1.358	1.087–1.896	0.039	1.268	0.953–1.698	0.195
TNM staging	1.994	1.205–2.945	0.008	2.051	1.325–3.152	0.005
Degree of differentiation	2.252	1.369–3.482	0.000	2.369	1.346–3.652	0.001
Lymphatic metastasis	2.169	1.286–3.385	0.002	2.289	1.269–4.215	0.001
Distant metastasis	1.815	1.135–3.252	0.026	1.585	0.989–2.652	0.085
FKBP10	3.395	1.654–5.224	0.000	3.255	1.598–4.892	0.000

## Data Availability

The data used to support the findings of this study are available from the corresponding author upon request.

## References

[1] Zhao J., Eyzaguirre E. (2019). Clear cell papillary renal cell carcinoma. *Archives of Pathology & Laboratory Medicine*.

[2] Akhtar M., Al-Bozom I. A., Al Hussain T. (2019). Papillary renal cell carcinoma (PRCC): an update. *Advances in Anatomic Pathology*.

[3] Linehan W. M., Ricketts C. J. (2019). The Cancer Genome Atlas of renal cell carcinoma: findings and clinical implications. *Nature Reviews Urology*.

[4] Wettersten H. I., Aboud O. A., Lara P. N., Weiss R. H. (2017). Metabolic reprogramming in clear cell renal cell carcinoma. *Nature Reviews Nephrology*.

[5] Wolf M. M., Kimryn Rathmell W., Beckermann K. E. (2020). Modeling clear cell renal cell carcinoma and therapeutic implications. *Oncogene*.

[6] Jonasch E., Walker C. L., Rathmell W. K. (2021). Clear cell renal cell carcinoma ontogeny and mechanisms of lethality. *Nature Reviews Nephrology*.

[7] Ascierto M. L., McMiller T. L., Berger A. E. (2016). The intratumoral balance between metabolic and immunologic gene expression is associated with anti-PD-1 response in patients with renal cell carcinoma. *Cancer Immunology Research*.

[8] Siegel R. L., Miller K. D., Fuchs H. E., Jemal A. (2022). Cancer statistics, 2022. *CA: A Cancer Journal for Clinicians*.

[9] Colwill K., Gräslund S. (2011). A roadmap to generate renewable protein binders to the human proteome. *Nature Methods*.

[10] Monsivais D., Vasquez Y. M., Chen F. (2021). Mass-spectrometry-based proteomic correlates of grade and stage reveal pathways and kinases associated with aggressive human cancers. *Oncogene*.

[11] Tang Z., Li C., Kang B., Gao G., Li C., Zhang Z. (2017). GEPIA: a web server for cancer and normal gene expression profiling and interactive analyses. *Nucleic Acids Research*.

The article "A Novel Biomarker, FKBP10, for Poor Prognosis Prediction in Patients with Clear Cell Renal Cell Carcinoma" was retracted in 2023. Reasons: signs of a paper mill; suspected computer-generated content; unreliable results or conclusions; concerns about the data.

[12] Ramadori G., Ioris R. M., Villanyi Z. (2020). FKBP10 regulates protein translation to sustain lung cancer growth. *Cell Reports*.

[13] Wang R. G., Zhang D., Zhao C. H., Wang Q., Qu H., He Q. (2020). FKBP10 functioned as a cancer-promoting factor mediates cell proliferation, invasion, and migration via regulating PI3K signaling pathway in stomach adenocarcinoma. *The Kaohsiung Journal of Medical Sciences*.

[14] Bonner J. M., Boulianne G. L. (2017). Diverse structures, functions and uses of FK506 binding proteins. *Cellular Signalling*.

[15] Ishikawa Y., Holden P., Bächinger H. P. (2017). Heat shock protein 47 and 65-kDa FK506-binding protein weakly but synergistically interact during collagen folding in the endoplasmic reticulum. *Journal of Biological Chemistry*.

[16] Duran I., Martin J. H., Weis M. A. (2017). A chaperone complex formed by HSP47, FKBP65, and BiP modulates telopeptide lysyl hydroxylation of type I procollagen. *Journal of Bone and Mineral Research*.

[17] Liang L., Zhao K., Zhu J. H., Chen G., Qin X. G., Chen J. Q. (2019). Comprehensive evaluation of FKBP10 expression and its prognostic potential in gastric cancer. *Oncology Reports*.

[18] Gong L. B., Zhang C., Yu R. X. (2020). FKBP10 acts as a new biomarker for prognosis and lymph node metastasis of gastric cancer by bioinformatics analysis and in vitro experiments. *OncoTargets and Therapy*.

[19] Ge Y., Xu A., Zhang M. (2017). FK506 binding protein 10 is overexpressed and promotes renal cell carcinoma. *Urologia Internationalis*.

[20] Xu W. H., Xu Y., Wang J. (2019). Prognostic value and immune infiltration of novel signatures in clear cell renal cell carcinoma microenvironment. *Aging (Albany NY)*.

[21] Knüppel L., Heinzelmann K., Lindner M. (2018). FK506-binding protein 10 (FKBP10) regulates lung fibroblast migration via collagen VI synthesis. *Respiratory Research*.

[22] Sun Z., Qin X., Fang J., Tang Y., Fan Y. (2021). Multi-omics analysis of the expression and prognosis for FKBP gene family in renal cancer. *Frontiers in Oncology*.

[23] Rahmani M., Nkwocha J., Hawkins E. (2018). Cotargeting BCL-2 and PI3K induces BAX-dependent mitochondrial apoptosis in AML cells. *Cancer Research*.

